The article "Droplet microfluidics: fundamentals and its advanced applications" was retracted in 2022. Reasons: plagiarism; overlap with other authors' work.

# Droplet microfluidics: fundamentals and its advanced applications

**DOI:** 10.1039/d0ra04566g

**Published:** 2020-07-23

**Authors:** Somayeh Sohrabi, Nour kassir, Mostafa Keshavarz Moraveji

**Affiliations:** Department of Chemical Engineering, Amirkabir University of Technology, Tehran Polytechnic Iran moraveji@aut.ac.ir

## Abstract

Droplet-based microfluidic systems have been shown to be compatible with many chemical and biological reagents and capable of performing a variety of operations that can be rendered programmable and reconfigurable. This platform has dimensional scaling benefits that have enabled controlled and rapid mixing of fluids in the droplet reactors, resulting in decreased reaction times. This, coupled with the precise generation and repeatability of droplet operations, has made the droplet-based microfluidic system a potent high throughput platform for biomedical research and applications. In addition to being used as micro-reactors ranging from the nano- to femtoliter (10^−15^ liters) range; droplet-based systems have also been used to directly synthesize particles and encapsulate many biological entities for biomedicine and biotechnology applications. For this, in the following article we will focus on the various droplet operations, as well as the numerous applications of the system and its future in many advanced scientific fields. Due to advantages of droplet-based systems, this technology has the potential to offer solutions to today's biomedical engineering challenges for advanced diagnostics and therapeutics.

## Abstract 2

Droplet-based microfluidic systems have been shown to be compatible with many chemical and biological reagents and capable of performing a variety of operations that can be rendered programmable and reconfigurable.

## 1. Introduction

The manipulation of fluids in channels with dimensions of tens of micro-meters, “microfluidics” has emerged as a distinct new field. The potential applications of microfluidics include a wide range from chemical synthesis and biological analysis to optics and information technology. Since the beginning of microfluidics, there has been a steady increase in the interest and development of devices for fluid flow at the microscale.^1,2^ Microfluidics is a multidisciplinary technology and neither it is limited nor belonging to an individual field. Clues for this originate from its applications in drug delivery, point of care diagnostic chips, organic synthesis^3^ and micro reactors.^4–6^ Typical laboratory operations can be performed in microfluidic systems with a fraction of the volume of reagents in significantly less time. Reagents can be significantly reduced from milliliters and microliters to nano-liters and femtoliters whereas hours of reaction time could be altered to mere seconds or even less.

Microfluidics is the science and technology of systems that process or manipulate small (10^−9^ to 10^−18^ liters) amounts of fluids, using channels with dimensions of tens to hundreds of micro-meters. The chemical analysis applications of microfluidics have some merits such as low cost, short times for analysis, the ability to use very small quantities of samples and reagents, and to carry out separations and detections with high resolution and sensitivity, and small footprints for the analytical devices.^7^ Microfluidics exploits both its most obvious characteristic, small size, and less obvious characteristics of fluids in micro-channels, such as laminar flow. It offers fundamentally new capabilities in the control of concentrations of molecules in space and time. As a technology, microfluidics offers so many advantages and so few disadvantages. However, for sure microfluidic technology will become a major theme in the analysis, and maybe synthesis of molecules. Microfluidic like other new technologies requires time and circumstances to be fully developed into a major new technology.

One subdivision of microfluidics is droplet-based microfluidics.^8,9^ unlike continuous flow systems, droplet-based systems use immiscible phases to create slugs or discrete volumes. Microfluidic systems are characterized by the low-Reynolds number flow regime which dictates that all fluid flow is essentially laminar. Continuous-flow based systems have exploited this phenomenon to create many novel micro-environments.^10^ For instance, a simple device has been created to study drosophila embryo development through local temperature control.^11^ Laminar flow behaviour also allows for the generation of precise concentration gradients that have been employed in the study of cell migration.^12^ Although continuous flow devices offer fine control over flow characteristics, scaling up is a challenge as the size of devices scales almost linearly with the number of parallel experiments.

Droplet microfluidics however, has the ability to perform a large number of reactions without increasing device size or complexity. In addition, recent discoveries have demonstrated that droplet microfluidic systems can perform simple Boolean logic functions, a critical step towards the realization of a microfluidic computer chip.^13–15^

Droplet-based microfluidics involves the generation and manipulation of discrete droplets inside micro-devices.^16,17^ This method produces highly monodisperse droplets in the nano-meter to micro-meter diameter range, at rates of up to twenty thousand per second.^18^ Due to high surface area to volume ratios at the microscale, heat and mass transfer times and diffusion distances are shorter, facilitating faster reaction times. Unlike in continuous-flow systems, droplet-based microfluidics allows for independent control of each droplet, thus generating micro-reactors that can be individually transported, mixed, and analysed.^19,20^ Since multiple identical micro-reactor units can be formed in a short time, parallel processing and experimentation can easily be achieved, allowing large data sets to be acquired efficiently. Droplet microfluidics also offers greater potential for increased throughput and scalability than continuous flow systems. In the past 5 years, several groups have used droplet microfluidics to form irregular particles,^21^ double emulsions,^22^ hollow microcapsules,^23^ and microbubbles.^24^ These particles can be used in a diverse range of applications, including the synthesis of biomolecules, drug delivery, and diagnostic testing.

We aim to provide an overview of the operations that have been developed to manipulate droplets and how such techniques can be applied to the chemical and biomedical engineering field. Recent reviews have focused on the theoretical basis^25^ and the chemical reactions that can be performed in droplets.^26^ We hope to illustrate the various methods and techniques that have been designed to provide precise control over parameters such as size, shape, and concentration inside the droplets. In addition, this review aims to illustrate the many uses of droplet-based microfluidic systems in real world biomedical applications.

## 2. Material of the device

In droplet-based microfluidics the choice of materials for the device microfabrication and fluid for droplet generation are two first design considerations. Poly(dimethyl) siloxane (PDMS), a relatively inexpensive and elastomeric polymer is the common for microfabrication. However, because PDMS is not stable in the presence of strong organic solvents or it is not compatible with some materials. Changes such as the swelling and deformation may occur and the use with greater solvent resistance such as glass,^27^ silicon,^28^ and thiolene can be suggested.

With the development of surface wettability and materials science, low energy consumption methods for controlling the wettability of liquids over surfaces have been possible. Among the methods, electro-wetting has superiorities such as fast response speed (several milliseconds), large switching range (several tens of degrees), outstanding durability (hundreds of thousands of switching cycles) and low energy consumption (10–100 μW). Fig. 1, represents the schematics of electrowetting on a dielectric (EWOD) from wetting to superwetting (inside the circle) with six basic fluid systems (outside the circle) based on three phases of water, oil and air. In all systems, there are a conductive droplet and an electrode covered with dielectric and hydrophobic layers. Most microfluidic devices are fabricated with W/A and O/W.^29^ Different W/O, O/W, and W/O/W emulsions can be developed by droplet- based microfluidics.

**Fig. 1:** From wetting to superwetting with different fluids.^29^

Teflon-like structure is both oleophobic and hydrophobic. Paper-based microfluidic systems are suitable for small-volume samples and their applicable detection perspectives are limited owing to the intrinsic cellulose matrix properties.^30^

The proper selection of material of the microfluidic system can be associated with application. The selection of glass is suggested for optical detection methods. However, with electronic detection methods, silicon and polymers are suitable. For electro-wetting, glass is the best option. For protein–protein interactions, PDMS is the best choice of material. For organ on chip applications, a wide selection of materials such as silicon, glass, PDMS and other polymers can be combined with hydrogels, biopolymers and additive manufactured scaffolding using proteins and the organ cells themselves. For bioprinting hydrogels, photocurable resins, and cells and the biopolymers are mostly used. In bioassay, the materials that inhibite enzymes should not be used in the microfabrication. For example, fused silica does not have a strong inhibition effect on PCR enzymes, but glass is a better option.^31^

## 3. The size of drop in microfluidic systems

Microfluidic flow is characterized by low Reynolds number (Re < 1) and the balance between interfacial tension and shearing force determines the droplet size. The ratio of the viscous stress to the interfacial tension is regarded as capillary number , where *μ*_C_ and *u*_C_ the velocity and dynamic viscosity of the contiguous phase. The surface tension at the rupturing trice (mN m^−1^) is*δ*. The lower the surface tension, the lower the droplet size and the higher the production frequency.^32^ Microfluidic flow is classified into continuous flow or segmented flow. The later is divided in to gas–liquid and liquid–liquid (droplet-based reactors). In continuous flow, the chemical composition can be adjusted by adding the reactants along the microfluidic system, but due to the parabolic velocity profile in laminar flow, the particle residence time is different, which can lead to polydispersity. However, the residence time distribution (RTD) in droplet-based systems is narrow and the coefficient of variance associated with droplet size is very low.^33^ There are three regimes in the droplet formation based on the capillary number of the continuous phase: squeezing or (Ca_c_ < 0.002), transient or cobbles flow (0.002 < Ca_c_ < 0.01), and dripping or drop flow (0.01 < Ca_c_ < 0.3).^34^ To have a complete understanding of the flow, it is common to construct, the flow map based on the Weber number  of the dispersed phase with respect to the We or Ca number of the continuous phase. Where, “*ρ*” and “*u*” are the density superficial velocity of the dispersed phase and *d* is the channel width.^35^ The microparticles with controlled size, shape, and monodispersity are popular in food processing, pharmaceuticals for drug delivery, cosmetics, tumor annihilation, synthesis of nanoparticles, enhancement of mixing reactions for chemical industries, creation of emulsions, crystallization of proteins, personal health care products and bubble generator.^34^ The channel geometry, channel aspect ratio and flow rate ratio affects the velocity, formation, length, volume, shape and size of drops.^32^ The effect of viscosity of the continuous phase on size and droplet generation rate have been studied.^36^ Contact and injection angle are also influential on the droplet size.^34^ Surfactants are amphiphilic molecules, *i.e.* with different groups having affinities for different immiscible phases (water/air, water/oil, oil/air.). This property pushes the molecules to the interface and the surface tension between the two phases is decreased.^37^ Thus, the addition of surfactants in droplet-based microfluidic system will not only decrease the droplets size, but also improves the stabilization of interfaces droplets. Moreover, the biocompatibility of the system and the exchange rate of molecules between droplets can be managed.

## 4. Micro-droplet formation methods

In droplet formations, there exist two immiscible phases, referred to as the continuous phase and dispersed phase. The discrimination between them is based on quantity. The first one is the medium in which droplets are generated and the second one is the droplet phase.^38^ the flow rate ratio of the continuous phase and dispersed phase, interfacial tension between two phases, and the geometry of the channels used for droplet generation can affect the size of the micro droplets.^39^ In general, the micro-droplet formation methods can be classified into passive and active. In active methods an external energy such as electric, magnetic, centrifugal is needed.^40^ Passive droplet formation methods are simple and common. The geometries of passive micro-droplet generation includes cross-flowing, flow focusing and co-flowing.

Working under low Reynold's numbers ensures the laminar flow in the droplet based microfluidics often.^41^ The coefficient of variation is usually used to provide a description of droplet size from the standard deviation. Each of the listed methods offer a way to generate microfluidic droplets in a controllable manner with appropriate variable management.

## 5. Micro-droplet manipulation

The interminable interest toward the droplet-based microfluidics leads to the development of devices with more control, manipulate, and functionalize droplets. Beyond several methods of droplet generation, operations performed on droplets include fission, fusion, sorting, and mixing of the droplet contents. In addition polymerization can change the droplet phase. Micro/nano particles, cells, proteins, and DNA encapsulation in core–shell structures have also been reported.

### 5.1. Droplet generation

The strength of droplet-based microfluidic systems originates from the production of uniform particles. Accordingly, fine control over the size, shape, and mono disparity of droplets is of the utmost importance. Several approaches have been developed for droplet generation with the same basic principles and materials. The emulsion created by two immiscible fluids such as water and oil can be considered a method for droplets generation.

#### 5.1.1. T-Junction

In the T-junction configuration, the inlet channel containing the intersection of the dispersed phase channel merges the continuous phase channel with the right angle.^42^ At the junction section, the interface can be observed between the two phases and as fluid passes the dispersed phase moves in the main channel. What lengthens the dispersed phase into the main channel is the shear forces that are caused by the continuous phase and the subsequent pressure gradient. The neck of the dispersed phase thins and eventually breaks the stream into a droplet (Fig. 2a). The fluid flow rates, the channel widths, and the relative viscosity between the two phases are influential factors on the droplet size in a T-junction. T-Junctions can have more than one inlet, and complex structures of them can be used in chemical reactions,^44^ and forming gas plugs^45^ and droplets of alternating composition.^46^

**Fig. 2:** Droplet formation with different mechanisms: (a) T junction (ref. 43), (b) capillary flow-focusing (ref. 43), and (c) di-electrophoresis-based generation (ref. 44).

#### 5.1.2. Flow-focusing

In the flow-focusing configuration, a narrow region forces the dispersed and continuous in the microfluidic device^47,48^ (Fig. 3a). In the flow-focusing due to the symmetrical shear exerted by the continuous phase on the dispersed phase, the generated droplets are stable. In addition to flow-focusing, the shear-focusing is also aimed to create a singular point of highest shear, which exists at the narrowest region of the nozzle.^49^ The continuous break-off of droplets from the fluid at maximum shear point confirms the formation of uniform droplets. The sizes of the droplets can decrease by increasing flow rates of the continuous phase. Moreover, as shown in (Fig. 2b), also increases the frequency of droplet generation rises by an increase in oil flowrates.^50^ There are different ways to devise flow focusing structures such as soft lithography or even the insertion of capillary sheathes into micro-devices. In the capillary design, the dispersed phase is injected through the capillary needle, and the continuous phase forms an outer shell around the central capillary.^23^ The orifice is the forced region for the two phases and the droplets are broken off downstream of the orifice (Fig. 3b)^51^ Flow focusing methods have also been used to generate microbubbles,^52^ multifunctional particles,^53,54^ ionic fluid emulsions,^55^ and double emulsions.^56^

**Fig. 3:** (a) Formation of water-in-silicone oil droplets using a flow focusing design with an embedded circular orifice. (b) Graph showing decreasing droplet size and increasing frequency of formation with increasing oil flow rate (ref. 48).

#### 5.1.3. DEP-driven droplet generation

Di-electrophoresis or DEP, can be used to generate uniform droplets by pulling the droplets from a fluid reservoir^57^ (Fig. 2c). It is different from electro-osmosis and other EHD processes because the fluid can be electrically neutral, and the force exerted on the uncharged fluid is caused by a non-uniform electric field.

#### 5.1.4. EWOD-driven droplet generation

EWOD devices can be fabricated as either a one or two plane device. In a two plane device the ground electrode is often placed on the top layer with the control electrodes on the bottom. Both layers include an insulating layer separating the droplets from the electrodes. Activation of the electrodes initiates fluid wetting of the channel and within tens of microseconds, the fluid begins to form a short liquid finger between the electrodes. The electrodes are then switched off, reverting the surface back to being hydrophobic. This causes the finger to break off from the reservoir, and form a droplet.

The size of the droplet is dependent on the electric field strength, frequency of the applied field, and width of the channel opening. For example, higher frequencies produce small droplets whereas lower frequencies generate larger droplets. Picoliter to femtoliter sized aqueous droplets have also been produced using EHD generation methods. One advantage of EHD generation is that no external pumps are required, allowing the system to become more compact and appealing for use in point-of-care devices.

### 5.2. Microbubble generation

In addition to liquid–liquid phase emulsions, gas–liquid dispersions have also been reported in microfluidic systems. Control over the size and volume fraction of microbubbles are critical for their applications.

A large number of methods have been developed for droplet generation, but due to the formatting of this review they cannot all be covered in detail presently. Droplet generation systems have been created using a variety of different methods of generation and control mechanisms including pressure,^58^ flowrates,^59^ viscosities,^60^ electrical,^61,62^ and centrifugal force.^63^ In addition, generation components have been parallelized to scale up droplet generation.^64,65^Table 1 provides a brief summary of the droplet size and generation frequency ranges of various droplet-based microfluidic systems, however it does reveal the wide range of capabilities of droplet microfluidics.^66^

**Table 1:** Size and frequency distributions for various droplet generation systems

	Geometry and material	Continuous phase	Size/μm	Frequency/Hz
Water in oil	Channel array in silicon^78^	Kerosene with monolaurate	21	∼5300 (est.)
	T-Junction in acrylated urethane^44^	Decane, tetradecane, and hexadecane with Span 80	10 to 35	20 to 80
	T-Junction in PMMA^45^	High oleic sunflower oil	100 to 350	10 to 2500
	T-Junction in PDMS^60^	C_14_F_12_ with (C_6_F_13_)(CH_2_)_2_OH	7.5 nl (plug flow)	2
	Shear-focusing in PDMS^52^	Oleic acid	13 to 35 (satellites <100 nm)	15–100
Oil in water	Channel array in silicon^78^	Water with SDS	22.5	∼5300 (est.)
	Sheath flow in glass caplllary^79^	Water with SDS	2 to 200	100 to 10 000
Gas in liquid	Flow-focusing in PDMS^83^	Water with Tween 20	10 to 1000	>100 000
	Shear-focusing in PDMS^86^	Water with phospholipids	5 to 50	>1 000 000
Liquid in air	DEP on hydrophobic insulator^62^	Air	10 pl	∼8 (est.)
	EWOD on hydrophobic insulator^32^	Air	∼700 nl	∼1 (est.)

### 5.3. Droplet fission

The advantages of using droplet microfluidics over continuous flow systems are its throughput, scalability, and its ability to run parallel experiments. Since each droplet can act as a vessel for reagents, by dividing the single droplet into two or more droplets, the experimental capacity can be straightforwardly scaled up. Therefore, droplet fission or splitting is a critical operation that can enhance the effectiveness of droplet-based microfluidic systems. In addition to increasing experimental throughput, droplet fission can also be used as a method to control the droplet content concentration.^67^

#### 5.3.1. Passive fission

Passive methods rely on the shear forces created by channel design to split the droplets at precise locations into controlled volumes without any components or forces. Droplet splitting has been performed with several channel designs including a T junction,^68^ branching channels,^69,70^ and with channel obstructions^71^ (Fig. 4a and b).

**Fig. 4:** (a) Bifurcating channel geometry used to halve droplets at each junction (ref. 70). (b) Pillar in channels demonstrates asymmetric fission of water-in-oil droplets (ref. 71). (c–e) Active fission of droplets using DEP through surface electrodes in EWOD system (ref. 72).

#### 5.3.2. Active fission

Once external force or electrical control plays role in the splitting mechanism, active fission occurs. Neither found in closed channels nor open surfaces, but between electrically addressable parallel plates, droplets are transported and fission occurred by EWOD. There is no specific channel patterns to guide the droplets moving and the travel path is dynamically determined through the electrode pads. The droplets are formed on a dielectric surface, which exists between the electrodes and a non-conductive substrate. Splitting is achieved when the surfaces near the opposite ends of a droplet are activated, and the surface central to the droplet is grounded. The activated regions will pull the droplet towards its respective ends, causing the droplet to pinch and divide in the middle. The controllable EWOD splitting of a droplet into two equal volumes has been demonstrated with EWOD^72^ (Fig. 4c–e).

### 5.4. Droplet fusion

Controlled coalescence of droplets is an important means of performing reactions within droplets. Reactions in droplets can be used for a number of applications, including the formation of particles, chemical synthesis, kinetics studies, or for the synthesis of biomolecules. For some reactions, it is critical for reagents to be kept separate until the proper conditions are available.

#### 5.4.1. Passive fusion

In passive droplet fusion, the location of droplet fusion is controlled by the channel design. Appropriate fusion depends on droplet frequency matching under high flow conditions. These challenges can be overcome by controlling the droplet generation frequency through adjusting the flowrate and channel geometry.^73^

#### 5.4.2. Active fusion

Active fusion of droplets has been achieved using EWOD and other electric-controlled methods.^74^ An electro coalescence of tightly packed droplets was performed within 100 ms with voltage as low as 1 V DC.^75^ Electrodes were placed parallel to the droplet channels and a range of AC and DC voltages were used to fuse droplets or cells.^76^ DEP has also been used as a method of droplet fusion.^77^ As long as the droplet composition is dielectrically distinct from its carrier fluid, DEP can be used to manipulate the droplet. Activation of electrodes adjacent to a droplet initiates droplet movement. By sequentially turning a series of electrodes on and off, the droplet can be guided toward another droplet until coalescence occurs.^78^ Researchers used a combination of an expanded channel configuration to bring two surfactant stabilized droplets close to one another, and parallel aligned electrodes to fuse the droplets.^79^

### 5.5. Mixing in droplets

The Peclet number (Pe = *uL*/*D*) is defined as the ratio between advection time and diffusion time, where *u* is the characteristic velocity, *L* the characteristic length and *D* the characteristic diffusion coefficient. In the domain where Re is small and Pe is large, mixing becomes difficult.^80^ Micromixer is an important tool required for carrying out and studying the kinetics of biological and chemical reactions. When dealing with fluids in the microscale, one major problem is being able to overcome interfacial forces and promote mixing between two fluid streams. Due to laminar flow conditions, when two fluid streams come into contact with each other, there is no turbulent mixing and the only mixing behaviour is diffusive. The same properties that allow adjacent miscible fluids to flow in distinct streams becomes a problem when one needs the fluids to mix. Although the diffusion distance is smaller, the time required to completely mix the two fluids is still long. Even inside droplets, the laminar flow conditions can be preserved and has led to the development of interesting biphasic particles. Continuous microfluidics is less efficient than droplet-based microfluidic system due to the slow mixing in microchannels.^80^ Smart channel configurations have been implemented to promote rapid internal mixing within droplets. Mixing in channels with serpentine pattern is very efficient, and the extent of mixing can easily be quantified with the length of the microchannels.^81^ Electro wetting based droplet devices have also developed mechanisms to rapidly mix the contents inside droplets. Hyunjung Lim *et al.* (2020) invented a dome-shaped chamber-based surface acoustic wave (DCSAW) device for the first time, which can be fabricated simply using a single adhesive tape and a drop of ultraviolet-curable material without soft lithography processes. As shown in Fig. 5 fluids A and B were injected into the inlets. By applying an RF signal to focused interdigital transducers (IDT) (F-IDTs), the concentrated acoustic energy was generated, and two fluids were mixed in the dome-shaped chamber. At an applied voltage of 20 V, mixing indices were higher than 0.9 at a total flow rate of 300 μL min^−1^.^82^

**Fig. 5:** (a) Schematic of dome-shaped chamber for micromixing using surface acoustic wave. (b) Cross sectional image of dome-shaped chamber on the line A–A′ depicted in (a). (c) Cross sectional image of fabricated dome-shaped chamber device for acoustic mixing.^82^

### 5.6. Droplet sorting

One of the key advantages of droplet microfluidics is the ability to generate unique droplets that can be transported and analysed individually. Sorting facilitates an array of functions including the isolation of droplets of interest, purification of synthesized samples and the segregation of heterogeneous mix of droplets. Additionally, sorting mechanisms enable individual control of single droplets out of a population.

Sorting can be divided into two types, passive and active. Passive sorting includes systems in which a bias is applied constantly to distinguish the species to be sorted. An active sorting system employs an increased level of complexity, but provides dynamic control over the bias and has more flexibility over the parameters it can sort. It needs to be noted that in passive sorting systems the bias and the sorting parameter is coupled; whereas in active systems the two need not be and thus allows active systems to sort droplets using a variety of characteristics such as particle content or functionality. More precisely, active sorting schemes involve both a mechanism to manipulate the movements of droplets and a method to detect the sorting criteria. Gravity and channel geometry has been employed to sort droplets passively by size and active sorting employs electrical control and has also been used as a mechanism to manipulate the droplets.

#### 5.6.1. Size-based sorting using channel geometry

An example of passive droplet sorting is the system designed by scientist.^83^ In this setup, the microfluidic channels are designed so that the flow stream of the continuous phase carries the smaller satellite droplets into a side channel, whereas the larger primary droplets flows through the main channel. Due to their smaller surface area, the satellite droplets are exposed to the flow projected from only the side branch whereas the larger droplet feels the higher velocity flow stream of the main channel. Since the satellite droplets are by products of the droplet generation process, sorting the droplets by size allows the sample to be purified. This concept was also applied to larger droplets. Gravity-driven size-based sorting. Another method that sorts droplets by size utilizes gravity. Researchers developed the mSOHSA—microfluidic sorting device with hydrodynamic separation amplification—which combines gravity-based sorting and channel design to purify perfluorocarbon droplets from a poly dispersed emulsion.^84^

#### 5.6.2. Dielectrophoresis-based sorting

An example of active sorting, DEP-based schemes allow manipulation of individual droplets, particles, or cells within microfluidic channels.^85,86^ Mazutis *et al.* (2013) has recently used DEP in a droplet-based microreactor for cell sorting. The cells expressing and secreting a target antibody are shown in grey and cells, which do not express a target antibody are indicated in orange. Cells are encapsulated in droplets with a fluorescent detection antibody. To produce secreted antibodies, cells are incubated off-chip and sorted according to the increased fluorescence signal from the localized packing of detection antibodies on the surface of the bead covered with capture and secretion antibodies (Fig. 6).

**Fig. 6:** DEP-based cell sorting.^85^

### 5.7. Electrowetting on dielectric (EWOD)-based sorting

Another example of active sorting mechanisms is EWOD-based droplet manipulation. As mentioned in the Droplet generation section, EWOD uses electrodes to change the interfacial energy between the droplet and the surface to cause droplet movement. This phenomenon can also be used to move droplets along a path. Scientist demonstrated sorting of droplets and its contents using this method by first separating two types of particles into opposite regions of a single droplet using electrophoresis, then splitting the droplet in half using EWOD.^87^

### 5.8. Phase change in droplet

Droplet-based microfluidics provides a robust platform for the manipulation of a variety of fluids and is capable of performing an array of operations and reactions. However, many biomedical applications require materials that are not liquid but in the form of solids or gels.^88^ Solid particles made from polymeric and biological materials are used in drug delivery^89,90^ and hydrogels^91^ are being studied for encapsulation of cells for implantation and drug studies. Many droplets based systems have been designed to create solid particles as well as hydrogel beads through different means.^92^

### 5.9. Photo-initiated polymerization

Photo-initiated polymerization uses light, usually UV to activate photo-initiators. The photo-initiators could then become a reactive radical. Radical polymerization then links the monomers and solidifies the droplet. Due to the use of optically clear polymer and glass, many microfluidic platforms are capable of integrating light sources into the set up to allow photo-initiated polymerization. Groups have demonstrated particle synthesis using this method with a variety of materials. More interestingly, novel particle shapes have been created using microfluidic platforms that cannot easily be made using traditional methods.

### 5.10. Catalyst-initiated polymerization

Unlike photo-initiated processes, this mechanism utilizes chemical species that trigger polymerization. Since the droplets are carried in the continuous phase, introducing the chemical trigger is not trivial. Two primary techniques have been developed to achieve this goal. First, the crosslinking agent, such as ions in the case of ionic crosslinking, could be contained in the continuous phase. After the generation of droplets, the cross linker diffuses into the droplet and causes the droplet to be solidified or gelled.^93,94^ scientist used this method to create capsules using a variety of materials including alginate, kappa carrageenan, and carboxymethylcellulose.^95^ The group was able to control the residence time in the chip and concentration of crosslinking agent in the continuous phase to create different types of particles. The process was terminated by putting the particles into a large volume of crosslinking agent free solution. Unlike traditional methods in which droplets are dropped into a polymerization solution, particles are synthesized *in situ* thus allowing continuous, high throughput processing.

### 5.11. Janus particles

The mechanisms used in the processes mentioned above all have equivalents in batch fabrication processes. However, synthesis techniques have been developed using droplet-based microfluidic systems to create particles that are difficult if not impossible to create macroscopically.^96^ These novel techniques take advantage of the unique properties of microfluidic platforms such as laminar flow and local control of flow conditions. These particular properties allow the research groups to create objects such as non-spherical particles, Janus droplets, and double emulsions.

## 6. Micro-droplet applications

Chemical and biological operations in cells, which are carried out in micron-sized spaces, are nature microfluidic examples. Droplet microfluidics offers the capability to compartmentalization and mimic reactions and molecular processes within individual droplets. With the device development in the transport and manipulation of droplets and particles, a number of opportunities can be found in combining these fluidic elements to carry out synthesis and functionalization of particles for biomedical applications. For this reason, droplet-based microfluidic platforms has a wide range of applications.

### 6.1. Control of chemical reactions

For applications ranging from protein expression to organic compound synthesis, performing reactions in the microscale conserves expensive and precious reagents, reduces exposure to hazardous chemicals, and allows multiple reactions to be carried out in highly parallelized experiments. In batch processes, there is high risk involved when performing exothermic reactions where large excess amounts of heat can be released. However, by scaling down the reaction in micro-reactors, parallel reactions can be performed with minimized risk. Reactions can also be done much quicker due to shorter diffusion and heat and mass transfer distances. Mixing inside micro-droplets also benefits from the internal vortex circulation directed by channel geometry.^97^

### 6.2. Therapeutic agent delivery

Due to the wide range of materials and methods available, the combination of polymers and other colloid particles can be used to alter drug release profiles, affect drug absorption rates, improve site specific targeting, and a number of other drug distribution characteristics. Current batch methods result in poly-disperse particles, thus microfluidic generation of micro-particles and microcapsules with reproducible size and femto-liter to nano-liter volume is a useful tool for therapeutic agent delivery. Control over particle size and minimization of the size distribution is important for the use of particles in the route of administration and controlled release of encapsulated materials such as drugs, dyes, enzymes, *etc.* The droplets can be filled with various hydrophilic or hydrophobic compounds and the capsule shell thickness can be altered to control compound release rates. Unlike diffusion limited continuous-flow micro-reactors, droplets with well-defined three dimensional boundaries allow rapid mixing and transport of reagents.^98^ Magnetic drug delivery is an active strategy that can be used to load nanoparticles in order to guide and accumulate them to tumor site by applying an external magnetic field.^99^

### 6.3. Biomedical imaging

Microbubbles have been used as ultrasound contrast agents in ultrasound imaging to develop the ability to image damaged tissues and serve as a tool for premature detection of diseases. The improved sensitivity and specificity of 2-D and 3-D ultrasound imaging can be achieved by increasing the reflection of the sound waves. The optimum reflectivity is size dependent and is observed with microbubbles 2–5 μm in diameter. Moreover, this size range is also suitable for passing through the capillaries in the lungs. The microbubbles increase sensitivity by enhancing the contrast in the image.^100^

### 6.4. Biomolecule synthesis

Biologists have long been on a quest to build artificial cells to understand the kinetics and biology behind life's most fundamental reactions. An artificial cell holds the advantage of having well-defined components that will allow scientists to study biological activities otherwise impossible. Micron-sized aqueous compartments that are capable of performing biological reactions are a first step to creating an artificial cell. Droplet microfluidics is not limited to the synthesis of particles and capsules, but can also be used for the synthesis of biological molecules such as protein and DNA.^101^ In droplet-based microfluidic generating a large number of cell-like compartments can be accomplished with controlled sizes, it enables the mimicking of Quorum sensing (QS)-type chemical communication. Niederholtmeyer *et al.* (2018) have fabricated artificial cells with a flow-focusing method. They showed that the artificial cells exchanged proteins with their neighbors. They prepared activator and reporter artificial cells containing gene templates for T3 RNA polymerase (RNAP) and for the T3 RNAP-driven synthesis of the TetR-sfGFP reporter, as well as a tetO array plasmid. The artificial cells containing both the activation and reporter constructs exhibited fluorescence as a function of density. The threshold density they observed was 400 artificial cells in 4.5 μL volume.^102^

### 6.5. Diagnostic chips

The main motivation behind the field of microfluidics is to create Lab-on-a-Chip devices based on the concept of the micro total analysis system (mTAS). The prospect of reducing processing time and consumption of reagents has prompted the development of many novel technologies aimed to replace traditional laboratory equipment. A large number of microfluidic devices have been designed to process biological reagents including cells, proteins and DNA.^103^ Droplet based platforms have the benefits of working on the microscale by having decreased diffusion distance, faster mixing, and laminar flow; but also the added advantage over continuous systems in that they can produce large numbers of micro-reactors to allow parallel processing while keeping each reactor independent and isolated. These unique properties have enabled a wide array of biochemical diagnostic assay to be performed using droplet-based microfluidic systems.^104^ Conventional detection methods are time-consuming and require expensive equipment, however, the developments of microfluidic chips for detection of fungal infections is very promising. Waseem Asghar *et al.* (2019) have developed an state-of-the-art immuno-based microfluidic device, which can rapidly detect and capture *Candida albicans* from phosphate-buffered saline (PBS) and human whole blood. So, fungal infection test can be executed in 1–2 hours instead of 2–10 days (Fig. 7).^105^

**Fig. 7:** The schematic comparison of conventional culture method and the microchip-based *C. albicans* detection.^105^

### 6.6. Drug discovery

The applications described previously have all dealt with the production or synthesis of materials in droplet-based microfluidic platforms. However, with the addition of optical and amperometric detection components such as mass spectroscopy, gel electrophoresis, and X-ray crystallography, droplet microfluidics has evolved into a platform with the potential for use in more sophisticated applications. Large diverse compound libraries can be quickly generated and screened in a single microfluidic device. This makes droplet-based microfluidics an ideal method for the discovery and study of new drug compounds.

### 6.7. Cell culture

One of the key advantages of droplet-based microfluidics is the ability to use droplets as incubators for single cells.^106^ According to literature review of the original 649 papers, Carla B. Goy *et al.* (2019) have found that cell culture is the most widespread application of the combination of hydrogel with droplet-based microfluidic system.^107^ Devices capable of generating thousands of droplets per second opens new ways characterize cell population, not only based on a specific marker measured at a specific time point but also based on cells' kinetic behaviour such as protein secretion, enzyme activity or proliferation. Recently, a surfactant-free method has been found to generate a stationary array of microscopic droplets for single-cell incubation.^108^ By droplet-based biopront (DBB) the controlled deposition of cells, growth factors, genes, drugs and biomaterials can be possible. However, a limited range of hydrogels including alginate, collagen, fibrin, methacrylated gelatin (GelMA) and polyethylene glycol (PEG), can been used in droplet-based bioprinting due to they or their crosslinkers can be ejected easily and the compatibility of their crosslinking mechanism with different droplet-based bioprinting modalities.^109^ Demirci's group fabricated coculture cancer models by bioprinting human ovarian cancer cells and fibroblasts in a controlled manner on Matrigel coated glass culture dish.^110^

### 6.8. Biological macromolecule characterization

#### 6.8.1. Protein crystallization

Droplet-based devices have also been used to investigate the conditions necessary for protein crystallization.^111^ The environment for protein crystallization can be adjusted by rapidly and continuously changing the flow rates of the input solutions. For long-term storage, protein crystals inside droplets can be transferred from microchannels to glass capillaries, and to obtain the diffraction pattern of the protein crystals, X-ray diffraction test can be performed.^112^

#### 6.8.2. Droplet-based PCR

Droplet-based microfluidic systems offer an outstanding technological platform for amplifying nucleic acids. In this regard, the most compelling application can be digital droplet PCR (ddPCR), which makes possible an extremely sensitive detection of specific nucleic acid sequences (down to the single copy level), and it originates from the statistical analysis of a large numbers of compartmentalized PCR reactions.^113,114^ Recently, in order to simplify the amplification process, alternative isothermal amplification scenarios have been developed. Such strategies include loop-mediated isothermal amplification (LAMP),^115,116^ rolling circle amplification (RCA)^117^ recombinase polymerase amplification (RPA)^118^ and exponential amplification reaction (EXPAR).^119^ Polymerase chain reaction (PCR) has been a vital tool in genomics and biological endeavours since its inception as it has greatly sped up production and analysis of DNA samples for a wide range of applications.^120^ Amongst these, LAMP has drawn the most attention due to its high sensitivity, high DNA product formation and reduced reaction times. In addition, using droplet LAMP (dLAMP) has a demonstrated benefit of enhanced inhibitor resistance compared to standard LAMP, and feasibility for point-of-care analysis.^121,122^

#### 6.8.3. DNA sequencing and barcoding

Multiple microfluidic systems, including droplet-based systems, have been used for DNA sequencing. A droplet-based microfluidic platform can analyse DNA molecules using a FRET ligation assay. The system is able to distinguish probes that perfectly complement a target molecule from the ones that are not complementary to the target molecule, even due to a single-base mismatch. Therefore, in its present form, the system enables rapid and inexpensive genotyping analysis. With an expanded probe set incorporating universal bases and containing all permutations of probes of a given length, it could be used for targets of arbitrary, unknown sequence, forming the basis for a fast and low-cost DNA sequencing platform.^123^

The monitoring of specific droplets amongst much larger droplet populations is a challenge when performing large-scale experimentation. The addition of small molecule- or quantum dot-based fluorophore mixtures to droplets can enable barcoding of a few thousand droplets at any given time, but is limited by spectral crosstalk in the condensed phase. In contrast, DNA barcoding, which involves the delivery of unique single DNA strands to each droplet, harvests an encoding capacity of 4^*n*^ (where *n* is the number of nucleotides in the DNA sequence), and is consequently practically unlimited in its ability to barcode exceptionally large droplet populations.^124^

### 6.9. Synthesis

Marco Faustini *et al.* (2013) have revealed a novel nanoliter droplet-based microfluidic strategy for continuous and ultra-fast synthesis of metal–organic framework (MOF) crystals and MOF core–shell structures. Representative MOF structures, such as HKUST-1, MOF-5, IRMOF-3, and UiO-66, were synthesized within a few minutes *via* solvothermal reactions with significantly faster kinetics than the conventional batch processes. Core-shell structures Co_3_BTC_2_@Ni_3_BTC_2_, MOF-5@diCH3-MOF-5, and Fe_3_O_4_@ZIF-8.^125^ Ioannis Lignos *et al.* (2018) have reported a combinatorial synthesis of highly luminescent and stable lead halide perovskite nanocrystals using a microfluidic platform, in which the typical flow rates were between 80 and 100 μL min^−1^ for the continuous phase and 0.1–50 μL min^−1^ for the precursors. Cs_*x*_FA_1−*x*_Pb(Br_1−*y*_I_*y*_)_3_ NCs has emission and absorption spectra between 690 and 780 nm.^126^ The synthesis of using a co-flowing microfluidic device has been reported. The hollow hydrogel microfibers is a carrier of microorganisms for mass-cultivation in an open system.^127^

## 7. Analytical methods for droplet characterization

The role of the quantitative analysis on the development of droplet-based systems is eminent. In this section, droplet characterization by methods including optical, electrochemical, mass spectrometry, Raman spectroscopy and absorption spectrometry have been addressed. The bright-field microscopy has studied not only the physical and biological behaviors of droplets,^128^ but also the kinetics for nucleation of protein crystals within droplets.^129^ Fluorescence microscopy, which is based on the excitation and emission of light from the molecule, is another dominant technique to quantify very low concentrations of biomolecules in droplets.^130^ As an example of fluorescence microscopy application, it can be referred to the measurement of enzyme due to the changes of fluorescence intensity inside the droplets with an Ar^+^ laser at a wavelength of 488 nm.^131^ Laser-induced fluorescence (LIF) can be applied for high-throughput screening and single-molecule detection in droplets.^132^ For instance, a droplet-based system has been used to detect fluorescence-labelled single DNA molecules by LIF.^133^ LED-IF systems, which are very compact and cheap, can be a good option for lab-on-chip applications and due to the single-wavelength nature of LEDs, they offer a high sensitivity and the maximum absorption wavelength can be tuned with test samples. As compared to the conventional LIF detections, six times lower LODs have been reported for LED-IF.^134^

Liu *et al.*^135^ developed a novel electrochemical method to measure the droplet characteristics on the basis of the chronoamperometric analysis of an electro-active compound in carrier phase. Once the droplets passed over the working electrode, their size and frequency can be attained by measuring the periodic variation of mass-transport limited produced current. Moreover, the droplet-based chips have been integrated with electrospray ionization-mass spectrometry (ESI-MS). Zhu *et al.*^136^ integrated droplet generation, droplet extraction and ESI emission on a single chip and used the hydrophilic tongue to extract the sample droplet while the oil flowed to the waste reservoir. In another study,^137^ a method for droplet injection in ESI-MS was introduced, by which the complex mixtures of reagents can be detected. As shown in Fig. 8, they directly coupled the droplet cartridge to a commercial nanospray emitter. Moreover, it also has the potential to be combined with other analytical techniques such as electrophoresis or high-performance liquid chromatography (HPLC) to enhance the capability of droplet-based systems.

**Fig. 8:** Schematic diagram showing the ESI-MS-based droplet analysis system.^137^

Hatakeyama *et al.*^138^ described the first use of matrix-assisted laser desorption ionization-mass spectrometry (MALDI-MS) for screening and optimizing reaction conditions in nanoliter-scale droplets. With the aid of fluorinated carrier, 30 nanoliter droplet reactors have been deposited on the MALDI plate. A group of 44 chemicals were screened against a specific substrate with a total substrate consumption of 20 μg in 2 μL solution.

A specific fluorescent labeling is mandatory for non-fluorescent analytes in laser-induced fluorescence (LIF) detection, prior to analysis. A label-free detection technique such as Raman spectroscopy is preferential and comes along with other advantages including the simultaneous detection of the multiple analytes, high throughput detection, high spatial resolution, and high sensitivity once they are coupled with surface-enhanced techniques.^139^ The earliest application of Raman spectroscopy in droplet system was reported by Cristobal *et al.* who took the advantage of high spatial resolution of Raman spectroscopy and mixed two non-fluorescent compounds inside droplets at different points along the microchannel.^140^

Absorption spectrometry offers a tool for study the kinetics of enzymatic reactions and measuring its parameters without the need to fluorescence information. Gielen *et al.*^141^ coupled single-point absorbance detection with a compartment-on-demand droplet platform to implement precise enzyme kinetics and inhibition analysis. As shown in Fig. 9, droplets were generated by moving the tubing up and down between the carrier phase and the aqueous phase from bottomless tubes under withdrawn mode, and droplet contents were quantified by transmittance *versus* time. They used a platform to study hydrolysis of a chromogenic substrate 4-nitrophenyl glucopyranoside by sweet almond β-glucosidase. Within 20 min, they measured the Michaelis–Menten kinetic parameters of the β-glucosidase. In addition, they also used a platform to measure the inhibition efficiency of conduritol B epoxide and 1-deoxynojirimycin targeting β-glucosidase.

**Fig. 9:** Schematic of the structure and sequential operation of a compartmented-on-demand droplet platform.^141^

## 8. Solutions of droplet-based microfluidics to biomedical challenges

Efficient multidrug delivery, which can be accomplished by Janus structure that enables loading two distinct materials or drugs into one vessel.^142^ The advantages of multi-drug delivery can be the efficacy of combination drug therapy through improving pharmacokinetics, temporally sequenced multi-drug release, and mitigating cytotoxicity to normal tissues while enhancing synergistic cytotoxicity in the tumor. Some common structure for co-drug delivery is shown in Fig. 10.^143^

**Fig. 10:** The schematics of multi-drug delivery systems.^143^

The pharmaceutical industry is currently suffers from unsustainable research and development (R&D) costs that forces it to alter how the development and approval of new drugs are pursued. Developing drug discovery using droplet-based microfluidics can solve such problems. In fact developing *in vitro* assays with which drugs could be examined, in the hope of increasing the predictability of a new drug before animal testing and human clinical trials. As an example, blood vessel-on-a-chip devices have already been used for the diagnosis of sickle cell disease in the clinic.^144^ Magnetically actuated droplet manipulation has also been applied for immunoassay. Immunoassays were accomplished to detect neonatal congenital hypothyroidism and analyzing umbilical-cord plasma sample. A typical example of magnetically actuated droplet manipulation in bioassay is for polymerase chain reaction (PCR).^145^

## 9. Commercial

Target applications of droplet-based microfluidics encompass cancer screening, microtoxicology, diagnostics, and sensing that benefit from the technological features of drop-based microfluidics.^146^ Commercial products of droplet-based microfluidics, which are associated with biological and healthcare problems includes 10x Genomics, Drop-seq and nucleic acid quantification *via* Droplet Digital™ PCR systems from Bio-Rad^126^ 10x Genomics and Bio-Rad QX200 is aimed at genome sequencing.^146^ Dolomite's drop merger chip^147^ is designed to fuse drops of a different composition. Fujifilm Dimatrix (DMP-2800) printer and Cluster Technology DeskViewer™ are two commercial Piezoelectric Drop-on-demand, which are developed for Bacterial cells to study cell-to-cell communications and Human liver tissue chips comprising of hepatocytes (HepG2) and HUVECs, respectively. RegenHU Ltd BioFactoryR is a commercial Micro-valve (Solenoid) is designed for 3D lung tissue comprising A549 cells, A.hy926 cells, and Matrigel™.^114^

## 10. Droplet microfluidics present and future

With new methods of fabrication, microfluidics has been able to exploit certain fundamental differences between the physical properties of fluids moving in large channels and those travelling though micro-metre scale channels. With special emphasis on the lab-on-a-chip devices, scientist have termed scaling relations, which associate or differentiate the macroscopic and microfluidic systems. Prior to be adapted as a major technology in future, microfluidics has some requisites. But it will live up to the hopes experienced at its conception. As a field, the problems it faces are those faced by most fields as they develop. The fact that microfluidics has not yet lived up to its early advertising is not a surprise, and the reasons for the rate at which it has developed are both characteristic of new technologies, and suggestive of areas in which to focus work in the future. Microfluidics being both a science and a technology offers great and even revolutionary new capabilities for the future. It is also in its initial stages, and a great deal of work needs to be done before it can be claimed to be more than an active field of academic research. However, the fundamentals of the field are very strong: much of the world's technology requires the manipulation of fluids, and extending these applications to small volumes, with accurate dynamic control over concentrations, while discovering and exploiting new phenomena occurring in fluids at the microscale level, must be very important.

For scale-up considerations, the use of parallel generators in a single chip is one way to achieve mass production to meet the industrial and commercial requirements. More than 12o droplet generators can be fabricated in a 4 cm × 4 cm chip to produce a throughput of 0.3 kg h^−1^ of monodisperse acrylic microspheres. The incorporation of hydrogel inside microfluidic chips widely contributed to the development of new biomedical, pharmaceutical and biotechnological systems. Microfluidic cell-culture systems and blood-vessel mimics on a chip can provide testing grounds for molecular robots that have medical functions to investigate the efficacy of drug transport to the cells. Future studies in biomedical imaging can evaluate the ways to measure the acoustic uniformity of mono-sized bubbles formed by flow-focusing. Step emulsification has potentials in the future utility in diagnostic applications such as ddPCR or isothermal and droplet generation methods can be useful for large-scale screening/selection applications. Raman spectroscopy is a promising technique for single-cell analysis. Thus, the combination of Raman spectroscopy with droplet-based microfluidics offers an exclusive opportunity to select cells for downstream single-cell manipulations, such as culturing cells and extracting DNA/RNA. Moreover, analytical detection techniques such as electrochemical detection, Raman spectroscopy, and mass spectrometry can be coupled to extend their application for droplet-based microfluidics.

## 11. Conclusion

This paper provides a comprehensive review of the field of “droplet” microfluidics and its applications. First flow characteristics and the parameters affecting the droplet size have investigated. Afterward, material selection in microfabrication have been studied. Moreover, the strategies toward microdroplet manipulation including droplet generation, sorting, fission, fusion, mixing, and polymerization have been presented. This nascent field has attracted a diverse group of researchers to study the fundamentals of two phase dynamics in micro-channels and also to develop novel solutions for biological and chemical applications that are superior to conventional techniques. Many examples are highlighted in this paper. Researchers in microelectromechanical systems (MEMS) have been developing novel microfabrication and surface treatment techniques to optimize droplet generation and manipulations in micro-device platforms. Microfluidic researchers have been focused on the control of droplet generation, droplet fission/fusion, mixing, and sorting to enable the high throughput analysis and synthesis conditions of large number of femto- to nanoliter volume droplets. Chemists are intrigued at being able to control reactions with precise concentrations and kinetic conditions and at the same time study them in large numbers. Biologists are seeing a rare opportunity to study bio-molecular and cellular events in cell-like environments and the notion of building “artificial cells” is much more realistic with the control that droplet microfluidics provides. Biomedical engineers are keen to developing “microsystems’’ with better robustness and reproducibility in order to enable new applications and industries at the interface of biomedicine and engineered devices/instruments. Some commercial products related to biological and healthcare problems are addressed. There are already companies that are developing droplet-based microfluidic products for the biomedical and biopharmaceutical industries.

Among the applications of droplet-based systems, some of them are eminent. Diagnostic chips have a very brilliant future. Microbubbles have been used as ultrasound contrast agents in ultrasound imaging. Droplet-based microfluidic system assists the chemical reactions to be done much quicker due to shorter diffusion and heat and mass transfer distances. The bright-field microscopy, Fluorescence microscopy, absorption spectrometry and electrospray ionization-mass spectrometry have been applied for droplet characterization. It is the belief of the authors that the rapid development of this field in just a few years and the vast amount of literature that is being generated points to a revolution in the field of Lab on a Chip that will continue for the next 5–10 years. This review paper is an attempt to capture a snapshot of the field and prosperous applications at this critical stage.

## Conflicts of interest

There are no conflicts to declare.

## Supplementary Material
